RETRACTED

# Deep Learning-Based Detection and Diagnosis of Subarachnoid Hemorrhage

**DOI:** 10.1155/2021/9639419

**Published:** 2021-11-22

**Authors:** Xiaohong Gou, Xuenong He

**Affiliations:** ^1^Department of Critical Care Medicine, Yongchuan Hospital, Chongqing Medical University, Yongchuan, Chongqing 402160, China; ^2^Chongqing Medical University, Department of Neurosurgery, Yongchuan, Chongqing 402160, China

## Abstract

Subarachnoid hemorrhage (SAH) is one of the critical and severe neurological diseases with high morbidity and mortality. Head computed tomography (CT) is among the preferred methods for the diagnosis of SAH, which is confirmed by CT showing high-density shadow in the subarachnoid space. Analysis of these images through a deep learning-based subarachnoid hemorrhage will reduce the approximate rate of misdiagnosis in general and missed diagnosis by clinicians in particular. Deep learning-based detection of subarachnoid hemorrhage mainly includes two tasks, i.e., subarachnoid hemorrhage classification and subarachnoid hemorrhage region segmentation. However, it is difficult to effectively judge reliability of the model and classify bleeding which is based on limited predictive probability of convolutional neural network output. Moreover, deep learning-based bleeding area segmentation requires a large amount of training data to be marked in advance and the large number of network parameters makes the model training unable to reach the optimal. To resolve these problems associated with existing models, Bayesian deep learning and neural network-based hybrid model is presented in this paper to estimate uncertainty and efficiently classify subarachnoid hemorrhage. Uncertainty estimation of the proposed model helps in judging whether the model's prediction is reliable or not. Additionally, it is used to guide clinicians to find the neglected subarachnoid hemorrhage area. In addition, a teacher-student mechanism deep learning model was designed to introduce observational uncertainty estimation for semisupervised learning of subarachnoid hemorrhage. Observation uncertainty estimation detects the uncertain bleeding areas in CT images and then selects areas with high reliability. Finally, it uses these unlabeled data for model training purposes as well.

## 1. Introduction

Subarachnoid hemorrhage (SAH) is a clinical syndrome which is caused by rupture of pathological blood vessels at the base or surface of brain and direct inflow of blood into the subarachnoid space, known as primary subarachnoid hemorrhage, which accounts for about 10% of acute stroke and is a very serious and common disease. The World Health Organization (WHO) survey shows that the incidence rate in China is about 2.0 per 100,000 people per year and there are reports that it is 6–20 per 100,000 people per year. These are also visible because of cerebral parenchyma, ventricular hemorrhage, epidural or subdural blood vessel rupture, and blood through the brain tissue into the subarachnoid space, known as secondary subarachnoid hemorrhage [1–5].

RETRACTED

Computed tomography (CT) is a medical imaging technique which has become a preferred method for initial diagnosis of subarachnoid hemorrhage due to its advantages of short scanning time and high sensitivity to blood. According to the characteristics of high-density lesions in the bleeding area in CT scan, radiologists can diagnose both the subarachnoid hemorrhage and the amount of hemorrhage in the patient's CT scan, thus providing reliable information for the development of corresponding intervention plans and methods. In addition, CT angiography (CTA) and magnetic resonance imaging (MRI) and other techniques are often used in the diagnosis of subarachnoid hemorrhage as a supplement to CT.

At present, imaging doctors need to examine a lot of CT image data every day and find lesions in layer-by-layer scans. The entire process requires a lot of energy. The huge amount of CT image scan data increases the risk of missed diagnosis and misdiagnosis. The imaging specialists have rich experience and can accurately diagnose subarachnoid hemorrhage in CT. However, due to limited energy, they cannot read a large amount of CT scan data. How to allocate expert power to the indistinguishable CT scan is the key to optimizing allocation of medical resources. For the estimation of patients' bleeding volume, imaging doctors often comment on subjective visual inspection or rough estimation methods to measure, and it is difficult to obtain accurate calculations in a short time [6–10].

In order to solve these problems, computer-aided analysis methods have received widespread attention and are widely used in different application areas, specifically hospital and industries. Computer-aided analysis is used to automatically or semiautomatically analyze image data by designing algorithms to obtain preliminary judgment results, thereby assisting imaging doctor in the next analysis. The imaging doctor conducts reexamination and verification on the preliminary results of the computer-assisted analysis, which greatly reduces workload. On the other hand, computer-aided analysis has the ability to screen out CT scans that are difficult to judge through massive amounts of data. Experienced experts can make more accurate diagnosis, which will improve the work efficiency of experts. For the quantification of subarachnoid hemorrhage, the computer can calculate the amount of bleeding in a very short time, providing an important quantitative index for the imaging doctor.

RETRACTED

To resolve these problems associated with existing models, Bayesian deep learning and neural network based hybrid model is presented in this paper to estimate uncertainty and efficiently classify subarachnoid hemorrhage. Uncertainty estimation of the proposed model helps in judging whether the model's prediction is reliable or not. Additionally, it is used to guide clinicians to find the neglected subarachnoid hemorrhage area. In addition, a teacher-student mechanism deep learning model was designed to introduce observational uncertainty estimation for semisupervised learning of subarachnoid hemorrhage. Observation uncertainty estimation detects the uncertain bleeding areas in CT images and then selects areas with high reliability. Finally, it uses these unlabeled data for model training purposes as well.

The remaining paper is arranged as follows: In Section 2, existing techniques, specifically those which are related to the problem under consideration in this paper, are discussed in detail.

## 2. Related Work

Subarachnoid hemorrhage is a subproblem of intracranial hemorrhage. Computer-aided analysis of intracranial hemorrhage can reduce the workload of imaging doctors, can reduce rate of missed diagnosis and misdiagnosis, and has great clinical application value. Therefore, a large number of researchers have proposed a variety of methods for computer-aided analysis. These methods are divided into two categories: intracranial hemorrhage subtype detection and intracranial hemorrhage region segmentation.

Liu et al. [11] designed a multistage preprocessing method and then extracted histograms and distance metrics as features and used support vector machines to classify CT slices. Ramteke and Khachane [12] used the nearest neighbor classifier to distinguish whether the CT slices include lesions based on statistical texture features. Shalokar et al. [13] calculated the gray-level cooccurrence matrix of CT slice images as features, then used genetic algorithms to select effective features, and finally used support vector machines for classification. These methods rely on human prior knowledge and require experts to design effective manual features. The proposal of deep learning [14] effectively fills the gap between low-level complex patterns and high-level semantic information, so that features at various levels can be automated end-to-end learning. Therefore, in recent years, most of the methods for detecting intracranial hemorrhage subtypes are based on deep learning technology.

Arbabshirani et al. [15] collected about 40,000 sets of data for training and about 10,000 sets of data for testing, which verified the effectiveness of the three-dimensional convolutional neural network in detecting intracranial hemorrhage. Chilamkurthy et al. [16] collected 290,000 sets of CT scan data from more than 20 hospital centers in India to train the model and also collected 20,000 (Qure25k) and 491 sets of CT (CQ500) scan data to verify the effectiveness of the model. He et al. used the convolutional residual network [17] to predict the occurrence probability of each subtype of intracranial hemorrhage in the CT scan layer and then used the random forest method [18] to combine the predicted probabilities of multiple scan layers to obtain the entire CT predictions of subtypes of intracranial hemorrhage scanned. Chang et al. [19] collected more than 10,000 sets of training data and 862 sets of test data. They designed a three-dimensional and two-dimensional hybrid convolutional neural network as the backbone network on the basis of Mask R-CNN [20]. Then it predicts the location of the intracranial hemorrhage area and its type. This method can detect the location of each subtype of bleeding in more detail.

RETRACTED

As for the segmentation of the bleeding area, it can be divided into the following categories: threshold-based methods, region-based methods, curve-deformation-based methods, brain atlas-based methods, machine learning-based methods, and deep learning-based methods. Based on the machine learning method, Li et al. [21] designed the distance feature to multiple landmark points, used the Bayesian decision framework to automatically segment the subarachnoid space area, and then used the support vector machine to classify the bleeding area in these areas. Based on deep learning methods, with the development of deep learning in image segmentation [22], many studies have also applied it to the segmentation task of intracranial hemorrhage. Manvel et al. [23] combined improved U-Net [24] and a dual-path network [25], which segmented the intracranial hemorrhage area from three perspectives and finally merged multiple separate training networks to predict the intracranial hemorrhage area. Islam et al. [26] extract output feature maps of VGG network and combine them into supercolumn features for intracranial hemorrhage segmentation.

## 3. Classification of Subarachnoid Hemorrhage Based on Bayesian Deep Network

In this section, we have introduced convolutional neural network for subarachnoid hemorrhage classification, which is obtained through network architecture search, and then two different techniques are proposed to assist in the judgment of network prediction. These methods are (i) uncertainty estimation based on Bayesian deep learning and (ii) region based on category activation map visualization that has a greater impact on prediction.

RETRACTED

### 3.1. Convolutional Neural Network

The classification performance of subarachnoid hemorrhage depends on the feature representation ability of convolutional neural network. Therefore, it is very important to select convolutional neural network with strong representation ability. With the successful application of AlexNet in the task of natural image classification, many studies focus on how to improve the performance of network, which is specifically reflected in improving the network structure, so deep learning network structures such as VGG, Inception, ResNet, ResNe Xt, and DenseNet have been developed. On the other hand, in order to achieve more powerful performance, the traditional approach is to increase the existing deep learning network in the following three aspects: depth, width, and input image resolution. However, these methods based on the manual design of the network structure and the unidimensional enlargement of the network are gradually replaced by network architecture search methods and statistical analysis methods.

The convolutional neural network selected in this chapter is based on the current excellent performance of EfficientNet. The model was chosen because EfficientNet was based on ImageNet large data set and network structure search method, and the performance was very good, so there is reason to believe that it has a stronger characterization ability. When the network model is scaled up to accommodate different computing resources, it has a more efficient mix of varying depth, width, and input resolution.

In this paper, the following changes are made on the basis of EfficientNet-B0 as shown in Table 1. The 2d dropout layer is added to output characteristic graph of each MBConv convolution module, which is considered to add regularization mode and also used for uncertainty estimation. Change the original resolution from 224 × 224 to 256 × 256.

### 3.2. Bayesian Deep Learning Model

Compared with nonprobabilistic deep learning networks, Bayesian deep learning considers the network parameters as a probability distribution instead of a certain number, so the probability distribution of the network under the conditions of a given data set can be obtained. In the inference stage, Bayesian deep learning can estimate statistics such as the mean and entropy of the predicted distribution, and obtaining the entropy used to measure uncertainty is the goal of this section. On the other hand, since the inference process of Bayesian deep learning cannot be solved by analytical methods, this chapter uses the practical Monte Carlo Dropout for approximate inference.

RETRACTED

To be specific, it is assumed that the parameter *ω* in the given deep learning network *f* is a random variable, and its initial prior distribution is *π*(*ω*). Under the condition of the given training dataset *D*, the posterior distribution of *ω* can be obtained by the following Bayes formula:

(1) $$\begin{array}{c} p\left(\omega |D\right)=\frac{f\left(D|\omega \right)•\pi \left(\omega \right)}{p\left(D\right)}. \end{array}$$

In order to obtain the posterior distribution, the integral term can be approximated by Monte Carlo sampling, or it can be directly approximated by variational inference using a simple and easy-to-calculate distribution.

The previous research proved that the variational inference based on Bernoulli distribution in the Gaussian process approximates the posterior distribution in a strict mathematical framework, which is equivalent to adding a Dropout layer to the neural network for training.

In other words, for the trained deep learning network with Dropout, its parameter distribution under the influence of Dropout *q*(*ω*) is similar to the postvalidation distribution of parameters under the Bayesian framework:

(2) $$\begin{array}{c} q\left(\omega \right)\approx p\left(\omega |D\right). \end{array}$$

Therefore, given a test intracranial CT image *I*, the probability distribution of its network prediction *y* can be calculated by Monte Carlo approximation:

(3) $$\begin{array}{c} p\left(y|I\right)\approx \frac{1}{T}\sum_{i=1}^{T}f\left(y|I,\;\omega_{i}\right), \end{array}$$

where *ω*_*i*_ ~ *q*(*ω*), that is, the weight obtained when Dropout is turned on. In addition, *T* represents the number of times. On the basis of the calculation result, this section measures the uncertainty by calculating the entropy value:

(4) $$\begin{array}{c} H\left(\overset{⟶}{p}\right)=-\sum_{c=1}^{C}p\left(y=c|I\right)\log\left(y=c|I\right). \end{array}$$

In summary, adding the Dropout layer to the training intracranial hemorrhage subtype classification network is no different from the Dropout regularization process. In the test phase, the Dropout layer needs to be turned on according to the working method of the training phase; that is, the probability of inactivation remains unchanged. Perform multiple forward propagations on the network to sample the network or network parameters, and then perform the abovementioned entropy calculation to obtain an estimate of uncertainty.

### 3.3. Category Activation Diagram

In classification of intracranial hemorrhage subtypes, in addition to the need for network output prediction results, humans often need to know which areas in input have a greater impact on the network's final prediction. Visualizing these areas can allow humans to try to understand the prediction of intracranial hemorrhage subtypes by deep learning networks. According to this, it is judged whether to sample the prediction result of the model. The category activation map or the category activation map based on gradient backpropagation is a commonly used visualization technique in deep learning. It is cleverly designed to obtain the area where the input has a greater impact on the output.

RETRACTED

The last layer of the convolutional layer in the deep learning network has the following characteristics: it contains abstract semantic information while retaining the maximum spatial location information. Therefore, visualizing the influence of the last layer of convolutional layer on the prediction output can reflect the degree of influence of the input area on the prediction and prediction. Assuming that the convolutional layer of the first *k* channel in the last layer of the network has a value of *f*_*k*_(*x*, *y*) at the position (*x*, *y*), the convolutional feature map is pooled by global average and then passed through the fully connected layer to get the logit probability output. For the first *c* category, the category activation image *M*_*c*_(*x*, *y*) can be obtained by the following calculation:

(5) $$\begin{array}{c} M_{c}\left(x,y\right)=\sum_{k}w_{k}^{c}f_{k}\left(x,y\right), \end{array}$$

where *w*_*k*_^*c*^ is the weight of the prediction output of the *c* category of the fully connected layer. If the position of the convolution feature map (*x*, *y*) contributes a lot to the category *c*, the value *f*_*k*_(*x*, *y*) on some channels *k* must be relatively large, and the corresponding *w*_*k*_^*c*^ must also be large. From this, we can get that *M*_*c*_(*x*, *y*) will have a higher response in these areas.

Since the deep learning network structure used in this paper meets this specific structure, it can be directly visualized in the abovementioned way. If the network structure does not conform to this specific form, the weight of the full connection of the structure can be replaced by the sum of the gradients.

## 4. Bleeding Region Segmentation Based on Teacher-Student Network

This section introduces, particularly in detail, teacher-student network that incorporates observational uncertainty. First explain the overall composition of the network structure and then introduce design of the loss function used for the estimation of observation uncertainty. Finally, show how to use uncertainty to weight the consistency regularization term.

### 4.1. Network Structure

As shown in Figure 1, the semisupervised segmentation method designed in this chapter includes two deep learning models with the same topology, namely, the teacher model and the student model.

RETRACTED

DPN92-Unet replaces its backbone network with a dual-path network on the basis of U-Net, which enhances the feature extraction capability. It has achieved preliminary results on the segmentation task of intracranial hemorrhage, so the deep learning model of the teacher-student model uses this structure as the basis. In order to meet the needs of subsequent tasks, DPN92-Unet needs to be modified in the following aspects: the convolutional layer with sigmoid activation function is added to the last layer of feature output map to observe the generated output of the uncertainty map. Dropout technology is added to the last layer of feature maps of the encoder and decoder of the network, so that the parameter disturbance of the model can be introduced.

In the training phase, the teacher model predicts the unlabeled data. This prediction will be used as the gold standard for unlabeled data to train the student model. Therefore, the accuracy and stability of the teacher model prediction becomes very important. In order to obtain a stable teacher model, the teacher model is not obtained through supervised learning and training updates, but is obtained on average through multiple student models at different training times. Specifically, the parameter *θ*_teach_ of the teacher model is obtained by the exponential moving average student model parameter *θ*_stu_:

(6) $$\begin{array}{c} \theta_{\text{teach}}≔\alpha \theta_{\text{teach}}+\left(1-\alpha \right)\theta_{\text{stu}}, \end{array}$$

where *α* is weight; this parameter is used to control the degree of influence of the current new student model parameter value on the average parameter value of the teacher model. The larger the *α*, the smaller the degree of influence, and vice versa.

The parameters of the student model are obtained by optimizing the objective function. Unlike supervised learning, the student model can obtain information from unlabeled data during the training process. This is achieved by introducing the regularization of the output consistency between the teacher model and the student model.

Formally speaking, suppose that a given available labeled data set *S*={(*x*, *y*)} and an unlabeled data set *U*={*x*}. $\hat{x}$ and $\tilde{x}$ represent the input *x* after different perturbations, where the input perturbation is pixel-level enhancement transformation or noise, which will not change the neighborhood structure of the space. The introduction of input disturbance is based on the thinking that a robust model should have similar predictions for two slightly disturbed inputs. In this way, the objective function of the student model can be expressed as

(7) $$\begin{array}{c} l\left(\omega_{\text{stu}}:\omega_{\text{teach}},S,U\right)=\sum_{\left(x,y\right)\in S}l_{\text{seg}}+\lambda_{\text{ucty}}\sum_{\left(x,y\right)\in S}l_{\text{ucty}}+\lambda_{\text{cons}}\sum_{x\in S}l_{\text{cons}}, \end{array}$$

where *l*_seg_, *l*_ucty_, and *l*_cons_ are the loss function of supervised segmentation, the regularization term of observation uncertainty, and the weighted consistency regularization term of observation uncertainty. And, *λ*_ucty_ and *λ*_cons_ are the weight values that increase with the training time, which respectively, control the importance of the uncertainty regularization term and the observation uncertainty weighted uniform regularization term on the training. They are set to 0 in the initial stage of training. This is because, in the initial stage of training, the weights of the student model are in the random stage. At this time, if the regularization term of the observation uncertainty is added, it is easy to make the training oscillate and it is difficult to converge. Similarly, the instability of the student model will also cause the teacher model's predictions to be unreliable. Increasing the consistency regularization too early will accumulate false predictions and cause the performance of the student model to decrease. The loss function of supervised segmentation uses a mixture of focal loss function and soft dice loss function, which is to solve the problem of category imbalance in the learning process. Specifically, the supervised segmentation loss function can be expressed as follows:

(8) $$\begin{array}{c} l_{\text{seg}}\left(p,y\right)=-{\left(1-p_{y}\right)}^{\gamma }\log\left(p_{y}\right)+\text{log}\left(\frac{2p•{\hat{y}}^{T}}{\left|p\right|+\left|\hat{y}\right|}\right), \end{array}$$

where *p* represents the segmentation probability prediction output by the student network, $\hat{y}$ is the one-hot vector representation of the gold standard *y*, and the parameter *γ* is the hyperparameter in the focal loss function, which is set to the recommended value *γ*=2 in the experiment.

RETRACTED

In the prediction stage, the teacher model is used as the final prediction model. In the experiment, it is found that the segmentation performance of the teacher model in the pre- and midterm training is better than that of the student model, but it gradually converges with the training of the student model. The difference between the teacher model and the student model becomes less obvious, and the performance between the two is about the same. However, because the teacher model is the average of multiple training periods of the student model, the robustness of the teacher model is reasonably considered stronger than the student model.

### 4.2. Uncertainty Loss Function

The uncertainty loss function is introduced as a regularization term, so that the student model can learn how to estimate the input observation uncertainty, because the teacher model is an average version of multiple student models. Therefore, the teacher model can also obtain this ability to estimate the uncertainty of the observation. Allowing the model to estimate the observation uncertainty has the following advantages: the model can be aware of the ambiguous areas in the input, such as fuzzy edges and noisy areas. These areas cause ambiguity and cannot accurately judge it. The model can have more opportunities to focus on certain areas rather than ambiguous areas. These ambiguous areas often make the labeling more likely to be wrong. Therefore, it is obviously more appropriate to introduce observational uncertainty to learn differently.

Intuitively, the relationship between prediction and uncertainty can be expressed as follows.

When the uncertainty is lower (the higher the confidence level), the penalty between correct prediction and wrong prediction is hugely different. The penalty for incorrect predictions needs to be significantly greater than for correct predictions.

On the other hand, when the uncertainty is higher (the confidence is lower), the penalty for correct prediction and wrong prediction is similar, and the penalty at this time is greater than the penalty for correct prediction when the uncertainty is low. This is because when a region itself has a large amount of noise introduced by observations, which makes it blurry, it is of little significance to judge whether it is correctly predicted. Penalties based on this idea will force the model to output correct predictions with low uncertainty (high confidence). At the same time, there is a certain degree of tolerance to correct those erroneous labels under high uncertainty.

The loss function used to learn to estimate the uncertainty of the observation is designed as follows:

(9) $$\begin{array}{c} l_{\text{ucty}}\left(\left(p,\psi \right),y\right)=-\left(1-\psi \right)\log\left(p_{y}\right)+\gamma \psi , \end{array}$$

where *p* and *ψ* are, respectively, the segmentation prediction map and the observation uncertainty estimation map output by the student model.

### 4.3. Uncertainty Weighted Consistency Regularization

When teacher model predicts unlabeled data correctly, then consistency regularization can be considered as a way to make the model training have more labeled data. This is because the consistency regularization makes the output of the student model and the teacher model on unlabeled data as consistent as possible. Therefore, it becomes very important to filter out reliable predictions from the predictions of the teacher model as the learning goal of the student model. Ambiguous image areas are difficult to clearly give a definite label (such as the position of the edge in subarachnoid hemorrhage), so it is more likely to cause incorrect labeling, and it is advisable to remove these fuzzy areas. In order to highlight the reliable area and the uniformly ambiguous area, the observation uncertainty estimation output by the teacher network is used for the weighted consistency loss function as follows:

(10) $$\begin{array}{c} l_{\text{cons}}\left(\left(p_{\text{stu}}\right),\left(p_{\text{teach}},\psi_{\text{teach}}\right)\right)=-\left(1-\psi_{\text{teach}}\right)p_{\text{stu}}-p_{\text{teach}}^{2}, \end{array}$$

where *p*_stu_ and *p*_teach_, respectively, represent the segmentation prediction probability of the student model and the teacher model for the same input. When the uncertainty of observation in a certain area is large, whether the output of the student model and that of the teacher model are consistent in these places will contribute little to the consistency loss function. Conversely, the consistency of the student model and the teacher model in a certain and reliable area will contribute a lot to the consistency loss function. Therefore, this makes the model pay more attention to certain and reliable areas and filter out ambiguity areas. The measurement of consistency uses the *L*_2_ generic number, which is to further reduce the influence of the teacher model's error prediction. Observation uncertainty estimation comes from the teacher model, which is to make this estimation stable.

RETRACTED

## 5. Experiments and Discussion

### 5.1. Evaluation on the Classification Model

Uncertainty estimation is a measure of the model's confidence in the input prediction. If the input CT image is unseen knowledge for the model and it is difficult to judge, the model will output a higher uncertainty. Conversely, if the model is confident about the current input CT image, the output will have lower uncertainty. Therefore, this characteristic of uncertainty can be used to screen the results of model predictions, and the classification performance of these predictions will have a higher accuracy rate.

Figure 2 shows the relationship between the confidence of each bleeding type in the test set and the performance indicators of each classification. The performance indicators include sensitivity, specificity, precision, F1 score, and accuracy. It can be seen that the classification performance is consistently improved with the increase in confidence, and the specificity and accuracy have always been at a higher score due to the existence of a large number of negative samples, which can eliminate the impact of the imbalance problem.

Figure 3 shows part of the CT images on the test set and the corresponding model prediction probability and uncertainty estimates. It can be seen that as the uncertainty decreases, the difficulty in judging intracranial hemorrhage and its subtypes from CT images gradually decreases. As the uncertainty decreases, the area of intraparenchymal hemorrhage gradually increases, and the performance is gradually obvious.

Figure 4 shows part of the CT images on the test set and their corresponding category activation maps. It can be seen that the category activation maps focus on some key areas. In addition to the bleeding area, they also focus on some task-related places and the edge area. In addition, because the category activation map is related to the category, more attention is paid to the task-related areas and the areas that are not related to the task are suppressed. The category activation map can determine whether the model is reliable or not and at the same time can guide humans to find the overlooked bleeding area.

Figure 5 compares the ROC curve and AUC value of ResNet and EfficientNet in the classification of subarachnoid hemorrhage. It can be seen that EfficientNet used in this chapter has more advantages in bleeding classification than ResNet, showing its excellent performance.

### 5.2. Evaluation on Bleeding Region Segmentation

Backbone network of the UctyMT model, which is proposed in this paper, is modified based on the DPN92-Unet network. A convolutional layer with a sigmoid activation function is added to the feature map of the last layer of DPN92-Unet to generate observation uncertainty estimates. In addition, the two-dimensional Dropout layer is placed on the feature map output by the last layer of the encoder and decoder to introduce the disturbance of the model parameters. We first train the model under supervised settings to verify the impact of each newly added module on the segmentation performance. Specifically, the models are compared under four-fold cross-validation. Each fold is trained for 100 rounds, and no unlabeled data is added to the training.

When the Dropout layer and uncertainty loss function are not added, DPN92-Unet only uses the segmentation supervision loss function for supervised training. When only the Dropout layer is added, the objective function still uses only the segmentation supervision loss function. When only the uncertainty loss function is added, the objective function is the superposition of the segmented supervision loss function and the uncertainty loss function, and the increase strategy of the weight value of the uncertainty loss function is the same as that used in UctyMT. Under the supervised training experiment, the performance of DPN92-Unet and its variant network on intracranial hemorrhage segmentation is shown in Table 2.

RETRACTED

In a supervised learning environment, the performance of DPN92-Unet using Dropout is slightly improved, and the loss of uncertainty does not improve the performance. In the semisupervised setting, UctyMT in both Dice and Jaccard gradually increases with the increase of unlabeled data. However, when the available unlabeled data exceed 30%, the performance of UctyMT increases slowly. UctyMT with all unlabeled data is 2.2% higher than DPN92-Unet without unlabeled data, Dice and 2.3% Jaccard, which proves the effectiveness of UctyMT in the use of unlabeled data.

In order to compare with other semisupervised segmentation methods, this chapter reproduces TCSE [27] and UA-MT [28] on intracranial hemorrhage segmentation. In addition, the experiment uses Mean Teacher [29] as a baseline model for segmentation tasks. For fair comparison and compatibility with two-dimensional input, the backbone networks of these models all use DPN92-Unet. These methods and UctyMT use 50% unlabeled data to train for 100 rounds until convergence. The experiment uses four segmentation performance indicators to quantitatively compare these methods, including slice Dice sparseness, slice sensitivity, patient Dice coefficient, and patient sensitivity. The cross-validation experiment results of each method using 50% unlabeled data are shown in Table 3.

Compared with the baseline Mean Teacher, TCSE slightly improves the segmentation performance by increasing the transformation consistency. Compared with TCSE, the slice Dice coefficient and sensitivity of UA-MT are increased by 0.74% and 0.62%, respectively, showing the effectiveness of removing unreliable regions. Among these methods, UctyMT in this chapter achieved the best segmentation performance in all indicators, achieving 78.12% and 78.58% in terms of average patient Dice and sensitivity, respectively. The slice Dice coefficient and sensitivity of UctyMT are 0.71% and 0.98% higher than that of UA-MT, respectively, indicating that, in the consistency regularization, the observation uncertainty mapping is more suitable for selecting the reliable region in the ambiguous data than the cognitive uncertainty.

## 6. Conclusions and Future Work

It is assumed that, through the preliminary judgment and screening capabilities of computer algorithms, workload of clinicians is reduced, thereby reducing the rate of missed diagnosis and misdiagnosis and achieving the goal of improving survival rate of patients. Focusing on the current fast-developing deep learning methods, this article applies these technologies to solve the key problems in the analysis of subarachnoid hemorrhage, while exploring new and efficient solutions. Specifically, this article focuses on two key issues in the analysis of subarachnoid hemorrhage: classification of subarachnoid hemorrhage and subarachnoid hemorrhage region segmentation. Most of the classification methods of subarachnoid hemorrhage are based on convolutional neural networks. In clinical applications, a single prediction probability is not enough to judge the reliability and safety of the model, and it cannot provide clinicians with more useful information. In response to these problems, this article is based on the current advanced deep classification model. We introduce the framework of Bayesian deep learning to estimate uncertainty, so that the model not only outputs the predicted probability, but also outputs the corresponding uncertainty estimate in the classification of subarachnoid hemorrhage. The uncertainty estimation of the model can effectively assist clinicians in screening reliable and high-confidence predictions, which makes the model safer and more reliable in clinical applications. In addition, the use of class activation map-based technology allows the model to visualize areas that have a greater impact on prediction, prompting clinicians to find areas of bleeding that are easy to overlook. However, the labeled data for subarachnoid hemorrhage segmentation is difficult to obtain, and a small amount of labeled data under supervised learning often makes deep learning overfit. In response to this problem, this paper introduces a semisupervised segmentation method in the subarachnoid hemorrhage region segmentation task. Based on the segmentation framework of teacher-student network, the performance of semisupervised segmentation of subarachnoid hemorrhage is improved by consistency regularization weighted by observation uncertainty.

RETRACTED

The proposed deep learning-based model should be enhanced such that the proposed model becomes an ideal solution for various other issues as well.

## Figures and Tables

**Figure 1:** Bleeding area segmentation network based on teacher-student network.

**Figure 2:** Relationship between classification indicators and confidence.

**Figure 3:** Prediction probability and uncertainty estimation.

**Figure 4:** Category activation diagram.

**Figure 5:** ROC curve and AUC value of ResNet and EfficientNet.

**Table 1:** EfficientNet network structure for bleeding classification.

Operation	Resolution	Channel	Layer
Conv3x3 & Dropout	226 × 226	32	1
MBConv1, k3x3, & Dropout	128 × 128	16	1
MBConv6, k3x3, & Dropout	128 × 128	24	2
MBConv6, k5x5, & Dropout	64 × 64	40	2
MBConv6, k3x3, & Dropout	32 × 32	80	3
MBConv6, k5x5, & Dropout	32 × 32	112	3
MBConv6, k5x5, & Dropout	16 × 16	192	4
MBConv6, k3x3, & Dropout	8 × 8	320	1
Conv1x1 & Pooling & FC	8 × 8	1280	1

**Table 2:** Performance of DPN92-Unet and its variant network.

Model	Dropout	Uncertainty loss	Unlabeled data (%)	Die	Jaccard
DPN92-Unet			0	86.8	83.9
DPN92-Unet	✔		0	87.2	84.5
DPN92-Unet		✔	0	87.0	84.0
UctyMT	✔	✔	10	87.4	84.7
UctyMT	✔	✔	20	88.1	85.4
UctyMT	✔	✔	30	88.7	86.0
UctyMT	✔	✔	50	89.0	86.2
UctyMT	✔	✔	100	89.1	86.2

**Table 3:** Comparison with other methods.

Method	Dice_s_	Sensitivity_s_	Dice_p_	Sensitivity_p_
Mean Teacher	87.4 ± 2.8	89.1 ± 1.9	75.2 ± 3.4	72.2 ± 3.7
TCSE	87.5 ± 2.2	89.3 ± 1.9	75.8 ± 2.9	73.7 ± 3.3
UA-MT	88.3 ± 2.3	89.9 ± 1.8	76.6 ± 3.0	74.9 ± 3.1
UctyMT	89.0 ± 1.9	90.9 ± 1.5	78.1 ± 2.3	78.6 ± 3.0

## Data Availability

The datasets used are available from the corresponding author on reasonable request.
